The article "Smart high-yield tomato cultivation: precision irrigation system using the Internet of Things" was retracted in 2025. Reason: concerns about the images.

# Smart high-yield tomato cultivation: precision irrigation system using the Internet of Things

**DOI:** 10.3389/fpls.2023.1239594

**Published:** 2023-08-22

**Authors:** Debabrata Singh, Anil Kumar Biswal, Debabrata Samanta, Vijendra Singh, Seifedine Kadry, Awais Khan, Yunyoung Nam

**Affiliations:** ^1^ Department of Computer Application (CA), Institute of Technical Education and Research (ITER), Siksha ‘O’Anusandhan (SOA) Deemed to be University, Bhubaneswar (BBSR), Odisha, India; ^2^ Department of Computer Science and Engineering (CSE), Institute of Technical Education and Research (ITER), Siksha ‘O’Anusandhan (SOA) Deemed to be University, Bhubaneswar (BBSR), Odisha, India; ^3^ Department of Computing and Information Technologies, RIT Kosovo (A.U.K), Rochester Institute of Technology – RIT Global, Kosovo, Albania; ^4^ School of Computer Science, University of Petroleum and Energy Studies, Dehradun, India; ^5^ Department of Applied Data Science, Noroff University College, Kristiansand, Norway; ^6^ Artificial Intelligence Research Center (AIRC), Ajman University, Ajman, United Arab Emirates; ^7^ Department of Electrical and Computer Engineering, Lebanese American University, Byblos, Lebanon; ^8^ MEU Research Unit, Middle East University, Amman, Jordan; ^9^ Department of ICT Convergence, Soonchunhyang University, Asan, Republic of Korea

**Keywords:** advanced network, Internet of Things (IoT), crop water requirement, smart agriculture, ml

## Abstract

The Internet of Things (IOT)-based smart farming promises ultrafast speeds and near real-time response. Precision farming enabled by the Internet of Things has the potential to boost efficiency and output while reducing water use. Therefore, IoT devices can aid farmers in keeping track crop health and development while also automating a variety of tasks (such as moisture level prediction, irrigation system, crop development, and nutrient levels). The IoT-based autonomous irrigation technique makes exact use of farmers’ time, money, and power. High crop yields can be achieved through consistent monitoring and sensing of crops utilizing a variety of IoT sensors to inform farmers of optimal harvest times. In this paper, a smart framework for growing tomatoes is developed, with influence from IoT devices or modules. With the help of IoT modules, we can forecast soil moisture levels and fine-tune the watering schedule. To further aid farmers, a smartphone app is currently in development that will provide them with crucial data on the health of their tomato crops. Large-scale experiments validate the proposed model’s ability to intelligently monitor the irrigation system, which contributes to higher tomato yields.

## 1 Introduction

In recent years, no other invention has generated as much excitement in the computing world as the Internet. Because of its tremendous strength and breadth of uses, it is virtually ubiquitous in every sector of human endeavor (Kumar et al., 2017; Poyen et al., 2020; Terence and Purushothaman, 2020). People and organizations have connected with amazing agility and convenience in recent years, thanks to a vast 5G network of wireless sensor networks (WSNs), healthcare services, cellphones, and various sorts of pervasive real-time monitoring systems (Lakshmiprabha and Govindaraju, 2019; Hassan et al., 2021). The human population is expanding at an alarming rate, but at the same time, pollution is slowly depleting the earth’s water and land supplies. Smart agriculture is seen as playing a crucial role in responding to these issues. Smart agriculture has the potential to vastly enhance both the agroecological setting and the yield and quality of agricultural products while simultaneously decreasing the need for harmful chemical fertilizers and pesticides (Zhang et al., 2022). The use of ICTs to automate and intelligently manage agricultural cultivation and production is central to the concept of “smart agriculture.” In particular, wireless communications play a significant role in the growth of agriculture, and each new generation of wireless communication technology propels farming toward a higher level of intelligence.

People and objects may connect in real-time thanks to the 5G network-based Internet of Things (IoT), which provides important services and value to millions of people across the world (Guevara et al., 2020; Biswal et al., 2021). 5G network-based IoT has developed organically into a gigantic technology platform. South America has initiated a yearly warm-season tomato yield that belongs to the Solanaceae family (Van Eck et al., 2019; Kumar et al., 2022).

Despite requiring high amounts of fertilizer, tomato is a popular or demanding plant due to its health significance to the whole world, with high levels of antioxidants such as carotenoid, lycopene, and vitamins C and A and phenolic compounds, which provide a wide range of health advantages for the consumers (Campestrini et al., 2019; Samanta et al., 2020; Chen P. et al., 2021). Tshiala and Olwoch reported that tomatoes have been used in food preparation throughout the world as fresh vegetables or as spices. It has a vital role in the Ethiopian marketing of vegetables (Guodaar et al., 2020; Biswas et al., 2021). The production of tomatoes was used as a job opportunity and as an income source for producers.

Nutrient and water supplies have a significant impact on tomato quality, and their highest water demand is quoted in an unpublished paper. Some poisonous elements and inorganic substances that are dangerous to people can demonstrate water quality (Sanjuan-Delm´as et al., 2020; Chen P. et al., 2021). This may be a problem for irrigation using municipal wastewater. Although municipal wastewaters have been applied as much as possible to irrigation, they contain comparatively maximum sodium quantities that can be accumulated with this wastewater and have toxic effects on plant soils during optimized irrigation (Jayalakshmi and Gomathi, 2019; Leuther et al., 2019; Casadei et al., 2021). The various types of crop growth models are extremely useful in optimizing irrigation practices which are based on physical or semi-empirical equations for simplification of the complex mechanism and also having many parameters in the process (Sanjuan-Delm´as et al., 2020). Because of its balance of simplicity, accuracy, and robustness, the AquaCrop model developed by the Food and Agriculture Organization (FAO) has provided a method for calculating crop yields and optimal irrigation scheduling for various crops in different climates. In the current real-time model, parameters like soil moisture (SM), crop cultivation, leaf area index (LAI), or canopy cover (CC) are collected using various remote sensing devices. As a result, this real-time cultivation process is an upgraded and fully dynamic version of the traditional models (Leuther et al., 2019; Chen P. et al., 2021).

A fast and dependable Internet connection is necessary for agricultural IoT devices to function. The current generation of mobile networks is failing due to insufficient connectivity in rural areas, and even in areas with high-speed access, failure occurs due to massive demand. According to a recent survey, nearly 80% of rural areas, even in the United Kingdom, are outside of the 4G range. The current degree of network access in rural areas is insufficient in most nations (Tang et al., 2021). In addition, in some developed countries, there are multiple farms with a large number of IoT devices and machines that require a constant reliable high-speed Internet connection to exchange a large amount of data, and the technologies of the current generation of mobile networks cannot cope with these demands (Singh et al., 2022). To fulfill these goals, many promising technologies, such as massive multiple-input multiple-output (MIMO), network slicing, and smaller cells, are needed to provide reliable connectivity over a larger distance. Therefore, the smart mobile network is well suited to support smart farming by enabling wide coverage, low-energy consumption, low-cost devices, and high spectrum efficiency.

Unfortunately, the IoT-based network’s usage of microwaves (MWs) as carriers limits its ability to cover wide areas. The introduction of small base stations spaced at roughly 250 m intervals over coverage regions that can be extended to any size allows for continuous connectivity, thanks to the small cell concept. In order to link the bigger areas, the related small towers can be placed everywhere (on lamp posts, in trees, on roofs, on tops of vehicles, etc.). Similar to 4G, this implementation makes use of the massive MIMO approach by equipping nodes with many antennas for sending and receiving data in order to increase the network’s capacity. On the other hand, huge MIMO makes signal interference more likely. Beamforming is used to increase the throughput of transmitted data and thereby solve this issue. Beamforming refers to an antenna’s capability of directing focused beams of radio waves at specific targets. An advanced Internet connection provides very high (MW) operating frequencies, and the accompanying high bandwidth makes it possible for larger and more rapid data transactions. In contrast to the static channels used by the 4G network, the cognitive radio approach used by the smart network allows for device-specific channel allocation.

In 2017, for the first time, the 5G RuralFirst project successfully planted and harvested a crop using autonomous tractors to sow seeds, drones to monitor crops, and machines to apply water, fertilizer, and pesticides. The entire procedure was carried out without the need for any laborers. Another initiative, Hands Free Hectare, claimed a successful harvest in 2018 (Al-Ghobari and Mohammad, 2011). With greater technological breakthroughs, 5G is projected to promote precision farming. As IoT-based network coverage grows, agricultural sector producers will benefit greatly, allowing them to manage farms, animals, and other assets from the comfort of their own homes, thanks to their big capacity, fast data speed, and low latency. Smart technology will help to advance IoT sensor connectivity to the next level, paving the way for unprecedented innovation in smart farming components. Implementing technology to automate, track, and monitor agricultural processes is a wise solution to the irrigation problem. The traditional irrigation method is fully automated by using IoT integration modules. However, with an advanced network on the horizon, smart agriculture will take off with lightning-fast data transfer.

To improve farm produce quality, smart farming combines traditional agronomic practices with the IoT. The application of new technology in agriculture can assist farmers in reducing labor and costs while increasing crop yield and production. To facilitate all of these agricultural benefits, the IoT includes a wide range of components under digital and automated technologies. So, IoT-based connectivity will vastly increase the impact due to low latency, high bandwidth, and support for many sensors communicating at the same time.

The IoT technology platform already helps to increase productivity and ensure proper resource utilization through precision agriculture. The implementation of IoT, on the other hand, will help to accelerate the entire process with machine-to-machine services. The real-time data transfer capabilities of the IoT module can aid in the rapid operation of these solutions, making decision-making quick, robust, data-oriented, and real-time. With an IoT-based network, these devices can send real-time data about the need for optimal irrigation, spoilt crops, and their location to follow-up machinery. Farmers can save time and money by harvesting crops quickly and effectively with automated irrigation for tomato crop cultivation.

The key contributions of this paper are as follows:

- An efficient IoT-based framework is proposed for tomato cultivation.
- Moisture levels in the soil are predicted with the help of IoT modules to optimize the irrigation system.
- A mobile application is also developed that can help farmers by providing useful information.

The remaining parts of the paper are arranged as follows. Section 2 discusses the literature review. Section 3 explains the things used for designing smart farming solutions. Section 4 details the proposed system and the methodology. The simulation setup and results analyses are described in Section 5. Section 6 concludes the paper.

## 2 Literature review

Chen et al. (2019) discussed the proper utilization of water for the growth of tomatoes by using the fuzzy neural network with a genetic algorithm (GA). It predicted the volume of irrigation based on the effect of greenhouse and the growth of crops (Guha et al., 2021). Rodríguez et al (Rodr´ıguez-Ortega et al., 2019). developed a soilless technique to yield tomato crops through the treatment of salinity. Here, the salinity treatment was specifically used to improve the production of vegetables and nutritional imbalance (psychological of plants) for crops. Zhai et al. (2015) proposed an idea for the cultivation of tomatoes using saline water and the blossom-end rot technique. Implementing these two yield methods enhanced the level of production.

In the study of Shao et al. (2014), two levels of irrigation techniques were designed for heavy rain shelters and drainage treatments for improving the productivity of crops. An optimum irrigation management technique was designed for yielding quality tomatoes through the proper arrangement of rain shelters (Keswani et al., 2020; Maroli et al., 2021; Mousavi et al., 2021). In the study of Gil et al. (2019), the smart grid system monitored the precision for irrigation of water on demand using IoT. The authors added desalination and solar energy processes in the agricultural system for efficient cultivation.

Krishna et al. (2017) designed a smart farming method for intelligent water-saving irrigation using the Raspberry Pi module and sensors. So, it automated the yielding of crops in a higher range that regulates through IoT modules. Qiu et al. (2020) implemented an in-depth process to collect phenotypic parameters for measuring the growth of tomatoes. This system precisely calculated the deficiency of water level and fertilizer with the help of a neural network algorithm for the growth cycle of tomato (Khamparia et al., 2020; Biswal et al., 2021). An intelligent irrigation system was defined as the water requirement for the yielding of tomatoes during a various range of climate states by Mason et al. (2019). In this study, smart irrigation was used in an adverse situation through proper integration of the IoT module, sensors, and connectionless environments (Chen M. et al., 2021).

In the agriculture industry, 4G/3G/NB-IoT wireless network technology is used to connect IoT-based smart devices for the purposes of data sharing, precise assessment, accurate calculation, etc (Dell’Uomo and Scarrone, 2002). Although the 3G/4G networking paradigm has shown much promise, there are still several obstacles that may prevent it from being used to its full potential in the agriculture sector. One of the main restraints is the available working space. Existing wireless networks do not reach out to rural areas or dense urban neighborhoods. Channel circumstances, resource allocation, fluctuating data rates, and handoff problems between diverse networks all make it difficult to facilitate quality of service (QoS) in 4G networks (Payaswini and Manjaiah, 2014; Payero et al., 2017). Mobile devices in this network have a short lifespan due to the utilization of many antennas and transmitters. Many modern agricultural sectors rely on battery-powered technologies like drones and robots, but these have limited usefulness in far-flung crop fields. The number of IoT devices used in smart farming, as well as the amount of research done on these devices, is growing rapidly, necessitating greater intelligence, speed, scalability, secure communication capabilities, and processing power to handle the numerous complex computational tasks and heavily utilized services. Having ultralow latency in addition to high connection is necessary for IoT devices to achieve quick performance and low costs.

The current 4G networks (LTE) are limited in their ability to enable such functionalities because they only permit connectivity through IP-based packet switching (Zhaogan et al., 2007). The shift to 5G cellular networks will eliminate these problems caused by previous generations of wireless technology. Due to advancements in 5G connectivity, farmers now have the option of remotely piloting a drone over extensive distances, either manually or via predetermined checkpoints (Faraci et al., 2018; Sinha and Dhanalakshmi, 2022). A farmer can get high-definition video streams and other critical sensory data and telemetry from drones in real time over the 5G cellular network, which is more efficient and reliable than previous-generation mobile networks (Bhattacharya and De, 2021). Due to 5G technology, drones will not need to carry a lot of computing power and instead can upload their data to the cloud, where it will be processed more quickly.

To demonstrate the importance of smart agriculture, Thilakarathne et al. (2023) show a cloud-enabled, low-cost sensorized Internet of Things platform for monitoring and automating processes related to a tomato plantation in a controlled indoor setting. We hope that the information gleaned from this study will be used as a foundation for advancing smart agriculture solutions that boost productivity and quality and pave the way for a more sustainable future.

Usman et al. (2022) present a 6G use case for plant health monitoring using a terahertz (THz)-signal-based integrated sensor and communication system. Precision agriculture is best understood as a smart management system with the capacity to track and regulate plant health and water levels on both a microscopic and a macro scale. The objective is to maximize output while minimizing waste of scarce resources. THz-based sensing technology, which can evaluate plant health on a cellular level, combined with wireless sensor networks installed within crops to monitor multiple variables while making intelligent decisions, could have significant implications for agriculture. A sustainable communication infrastructure that takes into account the needs of dispersed and adaptable agricultural settings is necessary for the integration and operation of such a macro–nano-sensor system.

## 3 Materials and methods

The growth and productivity of plants depend mainly on how much water is formed during the seedling phase. During this time, water demand has an important effect on crops, which have many environmental aspects like temperature, quality of soil, etc. The application of IoT in agriculture is limitless, which provides various intelligent devices to improve yielding performance and profit (Gomathy et al., 2020; Sivakumar et al., 2020). However, there are various issues with investing in smart cultivation and also difficulty in the development of agriculture-related IoT apps (Kamienski et al., 2019; Conesa et al., 2021).

a) Hardware unit:

The information will influence the development of IoT solutions for farming, and there is a need to select sensors to create the custom device that will collect data for the proposed solution (Althar and Samanta, 2021; Guha and Samanta, 2021; Zhang et al., 2021). However, the quality of the sensors has a crucial part in production which depends on the exactness of the collected data and its consistency.

b) Brain unit:

Smart agriculture should be used as data analytics for a design solution that will be helpful if yeomen cannot make sense of it, so there is a need to use powerful data analytics techniques and relate predictive algorithms and machine learning methods for collecting data.

c) Maintenance unit:

Hardware maintenance is a significant challenge for IoT-based agriculture, while the sensors are commonly used in the crop field. There are more chances for damaged sensors, which needs to be addressed by making a smart device that is robust and easy to sustain. Otherwise, it needs to be replaced with another sensor.

d) Mobility stage:

Smart farming applications can be remotely monitored through a smartphone or desktop computer for transmitting related yielding information to the owner (Maheswari et al., 2021; Mekala et al., 2021). The integration of devices should be autonomous and also cover enough wireless range to communicate and send data to the central server.

e) Infrastructure unit:

A solid and robust internal infrastructure needs to ensure that the intelligent cropping process performs well and securely handles the data load in it.

If the process disables the security, someone easily breaks the entire system and steals related data or controls intelligent devices.

### 3.1 Agricultural/crop production system

The cultivation model can be used to monitor or calculate the amount of native agricultural products, depending upon the cultivated area and supported by the decision support system (Nagarajan and Minu, 2018). **Figure 1** shows the agricultural/crop production prediction factors.

**Figure 1:** Crop-related and supply prediction factors.

The number of exports and imports of agricultural products can be derived from the prediction model of the National Statistical Office’s (NSO) statistics database as depicted in this section. The agricultural product crop and yielded area models are worked under the production of the smart agricultural prediction model, which evaluates the updated method as well as the predecessor observation method to reinterpret it.


(1) $$lnA_{x,t}=a_{0}+a_{1}lnRP_{x,t-1}+a_{2}lnRP_{y,t}+a_{3}lnA_{x,t-1}$$

where *A_x,t_* is seeding in *x* yield design at *t* year, *A_x,t_*_−1_ is seeding in *x* yield design at *t*−1 year, *RP_x,t_*_−1_ is the marketplace value in *x* yield design at *t*−1 year, and *RP_y,t_* is the market place value in *y* yield design at *t* year.


(2) $$Y\;D_{x,t}=b_{0}+b_{1}WT_{x,t}^{1}+b_{2}WT_{x,t}^{2}$$

where *Y D_x,t_* is the crop in *x* yield design at *t* year, *WT_x,t_* ^1^ is the weather (temperature) in *x* yield design at *t* year, and *WT_x,t_* ^2^ is the climate (amount of rainfall) in *x* yield design at *t* year.

The quantity of domestic products is the summation of agricultural products of all individual yield areas and each functional value of it (Gurunath et al., 2018; Mohanty et al., 2019; Benyezza et al., 2021). The agricultural product amount is the multiplication of the field with the crop model.

The demand method of the crop is the multiplication of the demand method per method in addition to the demands of the whole community. The resource purposes of agricultural products depend on export and import scenarios and other supporting factors, as depicted in **Figure 1**. The above equations must follow “Nerlove’s partial adjustment model,” and the regional weather information can help concede the prediction although there are some missing values (El-Zawily et al., 2019).

### 3.2 Challenges in the purpose system

Despite the many advantages that the 3G/4G networking paradigm offers, there are still several obstacles that prevent it from being used to its full potential in the agriculture industry. Space constraints pose serious problems. Current wireless networks are unable to reach more remote places or crowded metropolitan neighborhoods. Supporting the quality of service (QoS) in 4G networks is difficult due to channel conditions, resource allocation, varying data rates, and handoff problems between heterogeneous networks. Due to the heavy use of antennae and transmitters in this network, the lifespan of mobile devices is short. In order for Internet of Things devices to deliver quick performance at low prices, ultralow latency must be paired with a strong connection. Due to the limitations of IP-based packet switching connectivity on the existing 4G network (LTE), such features are now unavailable. These issues, which have plagued earlier generations of cellular networks, will be eradicated with the transition to IoT-based networks.

Due to its massive data capacity and speeds greater than 10 Gbps, IoT-based connection will be able to link billions of devices. For both download and upload speeds, 5G networks are expected to be up to 100 times faster than their 4G and 4G LTE predecessors. 5G can connect billions of devices due to its increased bandwidth, in addition to its large data capacity and speeds faster than 10 Gbps. The download and upload speeds of IoT-based networks will be up to 100 times faster than those of 4G and 4G LTE networks. Consequently, a 2-h movie that would take 6 min to download on 4G would take less than 4 s to download on an advanced network. Technical specifications for 5G are being developed by the International Telecommunication Union (ITU). The uplink peak data rate is 10 Gbps, and the downlink peak data rate is 20 Gbps per mobile station. Therefore, an IoT-enabled network is used for the Internet of Things-based smart irrigation system, which allows for remote monitoring of soil moisture and watering.

### 3.3 Mobile application

A mobile application is accessed by farmers on farms. Using this application, we can make predictions utilizing insight data and the collected cultivation insights data (Dhanush et al., 2017; Hota et al., 2020; Maheswari et al., 2021). The mobile application will provide crop-relevant information like crop health alerts, pest control, and warehouse inventory managing warnings as shown below. The key features of mobile applications are as follows:

- observing yield health facts (nutrient levels, pH levels, etc.) through the functionality of yield inspection (Ahmadi et al., 2019),
- the application of organizing fertilizer and insecticides for the farm (Kiryushin, 2019),
- automating the irrigation system and controlling water levels as well as soil health over the farm (Al-Ali et al., 2019; Li et al., 2020), and
- tracing yield records and checking warehouse details (bin inventories) (Quitaleg and Ortiz, 2020).

### 3.4 Impact of water quality on tomato yield

Tomato yield is a broad view that encompasses the interactions of various single-quality attributes. Irrigation water salinity enhanced tomato amounts, fruit thickness, soluble solids, total acid, vitamin C, and the sugar–acid ratio (Magán et al., 2008).

Fresh tomato yield, canopy diameter, fruit water content, tomato firmness, and calcium and nitrogen concentrations decreased as water salinity levels increased, whereas increasing salinity levels increased texture strength (Shao et al., 2014). In addition, saline water irrigation increased tomato fruit’s total soluble solids and acidity (pH) by 11.1% and 6.9%, respectively.

### 3.5 Role of the contactless IR sensors for tomato crop growth measurement

The contactless IR sensors are used to produce infrared radiation to measure the plant’s growth from its stem, whereas the radiation is converted into some amount of electricity and is less than 10 cm from the target. In the proposed system, sensors are placed more than 10 cm from the plant, which will measure growth by using a method based on the speculation of infrared energy. The IR sensors are fitted with infrared filters to avoid outside disturbing light. IR sensors are fitted to measure the thickness growth of tomato crops through the analog output voltage. The energy radiations of infrared sensors are transformed into distance data, which is not directly propositional to distance data.

## 4 Proposed system and methods

The evapotranspiration (ET) crop is described as the amount of water necessary for the perfect growth of various crops in connection with the lack of water by evapotranspiration which is discussed in this system. The demand for yielding waters refers to an optimally developed harvest, so that a consistent, disease-free crop is actively cultivated and completely sheltered. An advanced network can connect billions of devices due to its increased bandwidth, in addition to its large data capacity and speeds faster than 10 Gbps. The download and upload speeds of smart networks will be up to 100 times faster than those of 4G and 4G LTE networks. So, this method is advantageous in addition to IoT modules, which gives a perfect way to produce tomatoes in the seasonal and non-seasonal periods. The cultivation process is mainly influenced by the following situations like weather, yield type, and development stage of the harvest, which is depicted in **Figures 2**, **3**.

**Figure 2:** The proposed system for the smart irrigation of tomato yields.

**Figure 3:** Test scenario of the irrigation system.

The proposed system is integrated with the following components which are described below:

i. Arduino Uno microcontroller:

It is an open-source microcontroller that can be programmed by writing C or C++ code to control the overall system automation. After installing and programming the Arduino, it is ready to collect the number of inputs from IR moisture soil sensors and also provide a remote command to control the irrigation system. However, this microcontroller remotely controls the overall execution process.

ii. NIR-soil moisture sensor:

Soil moisture is a main attribute of soil and an important soil property that plays a vital role in a variety of farming activities, hydrological processes, and environmental concerns. A near-infrared (NIR) reflectance sensor is created for the calculation of moisture levels in the soil by implementing two light-emitting diodes (LEDs) of different wavelengths: one with a wavelength of 1,945 nm and a strong water absorption band and the other with a wavelength of 1,850 nm and a weak water absorption band. It is linked to an Arduino controller to record the moisture level of the soil. Accordingly, it gives instructions to the water controller for irrigation in the tomato cultivation land.

iii. Pinolex drip automatic water controller:

The smart flower irrigation timer is an efficient way to manage and control tomato crop irrigation needs. When you go on vacation or anywhere, an automatic water timer is set by the Arduino microcontroller, which is useful for watering tomato cultivation. It fits a 3/4-inch (19 mm) thread tap. It can water the plants regularly, even when no one is at home, and thus improve their survival rate.

iv. Wi-Fi access point:

A high-speed Ethernet wire links a router to an access point, which transforms a connection-oriented signal into a connectionless signal. Connectionless connectivity is typically the only available option for base stations, which use Wi-Fi to establish links with destination devices. As a result, the Wi-Fi service is linked to the 5G Internet, and it then provides a direct link with the end user to remotely monitor and control automatic irrigation as well as tomato crop cultivation.

### 4.1 Working principle of the model

The purpose model generally performs the operation in the following steps:

Step 1:

First of all, the NIR contactless sensor observes the moisture level of the soil. As a result, it is connected near the tomato plant to collect soil moisture. A field’s soil moisture status is critical for making planting, fertilizer application, and irrigation decisions.

Step 2:

Secondly, the moisture levels are observed through the Arduino Uno module, which is also linked with a Wi-Fi access point to send all the data to the mobile applications with the help of 5G technology. The 5G network helps to gather the moisture levels through the cloud service and automatically regulates the irrigation system.

Step 3:

When the moisture level is monitored through the mobile app, then the drip irrigation system is smartly controlled through the 5G-enabled IoT module (Arduino Uno microcontroller).

### 4.2 Evaporation and transpiration processes

Evaporation and transpiration happen at the same time, and there is no way to talk about them separately. The fraction of solar radiation that reaches the cropped soil surface is used to calculate evaporation. However, once the crop has matured to the point that it completely covers the soil surface, transpiration becomes the first process. IoT module sensors properly calculate the moisture level of the soil with the help of the calculation process of ET.

Evapotranspiration is commonly defined in mm/time, and water quantity lost from a cropped plane is defined in water depth units. Because 2 hectares has an area of 20,000 m^2^ and 2 mm equals 0.002 m, a loss of 2 mm of water corresponds to a loss of 10 m^3^ of water per hectare. Finally, 2 mm day^−1^ corresponds to 10 m^3^ ha^−1^ day^−l^.

The quantity of energy received per unit area can also be used to characterize water depths, with energy referring to the amount of heat or energy required to evaporate free water. The latent heat of evaporation (*λ*) varies with the temperature of water. At 21°C, for example, *λ* is approximately 2.50 MJ kg^−1^. To put it another way, 2.50 MJ is required to evaporate 2 kg or 0.002 m^3 of^ water.

### 4.3 Impact of weather on the yielding water requires reference crop evapotranspiration *ET_o_*

The main impact of weather information on crop water requirements is sunshine, temperature, moisture, and wind speed. The reference crop evapotranspiration defines the evaporation energy of the atmosphere (*ET_o_*). Reference crop evapotranspiration, also known as reference evapotranspiration, is the evapotranspiration rate from a reference surface that is not deficient in water and is expressed as *ET_o_*.

*ET_o_* values measured in distinct locations or climates are equivalent because they indicate identical reference surfaces. These variables influencing *ET_o_* can be parameters for climate, which can be measured using climate information. *ET_o_* intimates at a given location, the evaporating energy of the atmosphere.

In this research domain, different techniques are available for calculating *ET_o_*. It is tested either by an evapotranspiration pan or theoretically by using calculated weather information.

#### 4.3.1 Saucepan (pan) evaporation technique

The saucepan evaporation technique allows an environment to monitor the combined influence of temperature, moisture, wind speed, and sunlight on the reference yield evapotranspiration *ET_o_*. The various evaporation pans are class A evaporation pan and Sunken Colorado pan. The evaporation saucepan is used in the following equation:


(3) $$ET_{o}=K_{pan}\times E_{pan}$$

where *K_pan_* is the pan coefficient, *E_pan_* is the pan evaporation, and *ET_o_* is the reference yield evapotranspiration.

#### 4.3.2 Blaney–Criddle technique

The Blaney–Criddle method is a theoretical technique to determine the reference yield evapotranspiration *ET_o_*, and more literary techniques have been used, but many of them were locally calculated. If the process is accessed locally, if it is available or if local procedures are not available, then the theoretical method is used for the calculation.


(4) $$ET_{o}=P\left(0.46T_{mean}+8\right)$$

(5) $$\begin{array}{l} T_{max}=\frac{\sum_{month}\left(max\right)}{N_{days}{\;}_{/month}}\\ T_{min}=\frac{\sum_{month}\left(min\right)}{N_{days}{\;}_{/month}}\\ T_{mean}=\frac{T_{max}+T_{min}}{2} \end{array}$$

Where *ET_o_* = 1 month of average period,

*T_mean_* = regular temperature, and

*P* = regular proportion of yearly day time periods.

### 4.4 Impact of yield type on yield water requires *K_c_*

The single crop coefficient *K_c_* plays a significant role in crop characteristics as well as the averaged effects of soil evaporation. Average crop coefficients are more relevant and convenient than *K_c_* computed on a daily time step using a separate crop and soil coefficient for normal irrigation planning and management, development of basic irrigation schedules, and most hydrologic water balance studies (Farg et al., 2012). The impact of yield type on the yielding water requires dealing with the yield type and the development yield stage on water needs. The field is harvested between the relationship of reference grown yield and grown yield.


(6) $$ET_{{\;}_{Y\;ield}}=ET_{o}\times K_{c}$$

where *ET_Yield_* = yield evapotranspiration process (month/day), *K_c_* = yield influence, and *ET_o_* = reference evapotranspiration. Here, *ET_Yield_* and *ET_o_* are stated in equal units in month/day.

#### 4.4.1 Manipulation of the overall growing stage

From the beginning of transplantation to the last day, the overall growing stage of the crop is determined. It is primarily influenced by the following:

- the various harvest and its multiplicity,
- the condition of the weather, and
- the different stages of planting on the field.

#### 4.4.2 Manipulation of growth stages

The manipulation of the overall growing stages of yield is divided into four stages:

- the analysis of the yield first stage,
- the observation of the yield development stage in a field,
- the mid-time cultivation stage, and
- the late-time growth stage of the crop.

### 4.5 Different steps of estimation of the crop water requirement

The analysis of the requirement of aquatic crops *ET_crop_* is evaluated as:


(7) $$ET_{{\;}_{crop}}=ET_{o}\times K_{c}$$

#### 4.5.1 Yield of water quantity requirement of tomatoes

**Table 1** shows the given details of the crop.

**Table 1:** The given details of the crop.

Month (mm)	November	December–January	February	March	April	May
*ET_o_* (mm/day of crop)	5.0	4.5–4.0	5.0	5.8	6.3	6.8
Moisture state	Medium state	(60%)	–	–	–	–
Wind speed	Medium state	(3 m/s)	–	–	–	–
The growing interval (from the period of sowing): 150 days						
The specific date of planting: 1 February (direct sowing)						

This symbol means null or empty.

*Method of calculation:*

Step 1: The distinct growth stages of crop estimation are considered (see **Table 2**).

**Table 2:** The distinct growth stages of crop estimation.

Yield type	Final growing session (days)	Yield starting stage	Yield growing stage	Mid-time stage of yield	Late-time stage of yield
Tomatoes	150	35	40	50	25

Step 2: The month-wise tomato crop’s growth stages are observed (see **Table 3**).

**Table 3:** Crop: tomato planting date: 1 November.

Month (mm)	November	December	January		February	March	April	May
*ET_O_* (mm/day of crop)	5.0	4.5	4.0		5.0	5.8	6.3	6.8
Growth stages	Initial crop and development		Mid-time stage			Last session		
Crop sowing date				1 November				
Starting stage of the crop, 35 days				1 November–5 December				
Development stage of the crop, 40 days				6 December–15 January				
Mid-time stage of growth, 50 days				16 January–5 February				
Late–time stage of growth, 25 days				6 February–30 March				
Last day of crop growth				31 March				

Step 3: The *K_c_* factor for each of the four stages is estimated as (López-López et al., 2014):

*K_c_*, the starting stage of the crop = 0.45

*K_c_*, the development stage of the crop = 0.75

*K_c_*, the mid–time stage of the crop = 1.15

*K_c_*, the late–time stage of the crop = 0.8

**Table 4** shows the *K_c_* values.


$$\begin{array}{l} Nov-K_{c}:Nov=0.45Dec-5day:Kc=0.4525days:Kc=0.75\\ Dec-K_{c}:K_{c}=\frac{5}{30}0.45+\frac{25}{30}0.75=0.07+0.62=0.69≃0.7\\ Jan-15days:K_{c}=0.75\;15days:K_{c}=1.15,\\ Jan:K_{c}=\frac{15}{30}0.75+\frac{15}{30}1.15=0.38+0.58=0.96≃0.95\\ Thus,K_{c}-Jan=0.95,Feb-K_{c}=0.95,Mar-5days:K_{c}=1.1525days:\\ K_{c}=0.80\\ K_{c}:Mar=\frac{5}{30}1.15+\frac{25}{30}0.80=0.19+0.67=0.86≃0.85 \end{array}$$

**Table 4:** The water requirement for the complete growing time of tomato crop is 638 mm.

Month (mm)	November	December	January	February	March	April	May
ET_o_							
(mm/day of crop)	5.0	4.5	4.0	5.0	5.8	6.3	6.8
Growth stages	Initial crop and development		Mid-time stage		Last session		
*K_c_* per month	0.45	0.70	0.95	1.15	0.85		
ET_o_							
(mm/day of crop)	2.25	3.15	3.8	5.57	4.93		
ET_o_							
(mm/month of crop)	60	84	143	200	151		

Step 4:

**Table 4** shows the crop water requirement calculated on a monthly basis.


Nov = 5.0×0.45 = 2.25 mm/days

Dec = 4.5×0.70 = 3.15 mm/days

Jan = 4.0×0.95 = 3.8 mm/days

Feb = 5.0×1.15 = 5.75 mm/days

Mar = 5.8×0.85 = 4.93 mm/days

Step 5: Calculation of crop water requirement monthly.

Every month is supposed to have 30 days.


Nov=ET yield=30×2.02=60 mm/month

Dec=ET yield=30×2.8=84 mm

Jan=ET yield= 30×4.75=143 mm

Feb=ET yield=30×6.67=200 mm

Mar=ET yield=30×5.04=151 mm

**Table 4** shows the water requirement for the complete growing time of tomato crop, which is 638 mm.

## 5 Simulation setup and results analysis

In the proposed system, the related experimental data are received through the installed soil moisture and humidity sensor from the tomato crop field. The NIR REES52 Soil Sensor is used to collect the percentage of moisture in the soil. Based on this, an irrigation process is automated with a developed mobile application which is depicted in **Figure 4**. By using this app, the status of soil moisture and the growth of plants can be dynamically observed, and the irrigation method can also be controlled. Similarly, the plant growth parameters like maximum height, width, and diameter of the stem of the tomato plant are measured using an infrared sensor. This is tested in a regional area 28 m in length and 7 m in width, but the experimental site is portioned into two rows, and tomatoes are planted 4 m in length and 1.2 m in width zone. On the other hand, 50-cm-high PVC plates are applied for separation from communities, and a 50-cm row spacing is followed for the plantation of tomatoes. Data are captured continuously from the field of cultivation. The fog nodes are implemented for sensing data in the area of cultivation. The overall implementation of the proposed work is depicted in **Figure 5**.

**Figure 4:** Smart Irrigation Mobile App System. **(A)** App interface for monitoring various options. **(B)** Overview of various status of sensors. **(C)** Map of cultivation area. **(D)** Monitor soil moisture and crop status.

**Figure 5:** Overall Implementation of Irrigation System in the Field. **(A)** Irrigation pipe setup in between crops. **(B)** Automated water pump setup machine. **(C)** Drip irrigation in single row view. **(D)** Drip irrigation in a double row view.

The cultivation time to the collection period is from 1 November 2020 to 18 April 2021, as depicted in **Figure 6**, but it is drawn from the above data (**Table 4**), which is defined in step 5. The cultivation of the tomato growth period is evaluated as the crop sowing period to seedling period (November 1 to December 5), the development stage of the crop period (December 6 to January 15), the mid-time stage (flowering) of the growth period (January 16 to February 5), and the late-time stage of growth (fruiting and mature picking) period (February 6 to March 30). The analysis of irrigation data for tomato cropping depends on the relevant factor of the soil moisture sensor at 22 cm depth. This measure predicts the volume of irrigation.

**Figure 6:** Plot denotes the effect of **(A)** tomato yield on crop water requiring *K_c_* per month and **(B)** weather on crop water requiring *ET_o_*.

By the observation of moisture level from the above, **Table 5** shows a dynamic way of the automatic required level of irrigation for tomato cultivation (**Figure 7**).

**Table 5:** This is a calculated 41-day tabular record representation from the growing interval of 150 days after transplanting and also the percentage of soil moisture.

Days after transplanting	Percentage (%) of soil moisture	Days after transplanting	Percentage (%) of soil moisture
29	100	98	53
32	87	101	51
35	63	104	49
38	37	107	48
41	23	110	45
44	18	113	43
47	27	116	46
50	42	119	47
53	57	122	50
56	35	125	48
59	67	128	46
62	70	131	44
65	61	134	43
68	54	137	47
71	48	140	46
74	42	143	47
77	40	146	48
80	41	150	49
83	45		
86	50		
89	54		
92	56		
95	57		

**Figure 7:** The daily soil moisture percentage (%) during the experiment.

**Table 6** shows a feature-wise comparison of this paper with the existing literature. The existing work has been mostly considered under normal cultivation methods. However, in the proposed work, it is found that 5G technology is integrated with the IoT module. As a result, the irrigation system is working intelligently for the cultivation.

**Table 6:** Comparison of the proposed technique with the existing techniques.

Model	Approach	Data	Objective	Advantages	Limitations
Proposed precision irrigation system using the IoT-based model and mobile app	The 5G-enabled IoT-based model is used to provide precision irrigation and fast communication between various nodes.	Moisture level and crop coefficient (*K_c_*) are followed for the smart irrigation system.	Smartly cultivate tomato in the regional field with the help of IoT-based technology.	Through 5G technology and a mobile app, it can control the operation of the drip irrigation system remotely.	Energy conservation of the IoT module with a suitable communication protocol and also applicable to other crops will be designed in the near future.
Genetic optimization T-S fuzzy neural network model (Chen et al., 2019)	The modified genetic algorithm is used to optimize the weights and thresholds of the T-S fuzzy neural network. Finally, the genetic optimization T-S fuzzy neural network is utilized to simulate and estimate the irrigation volume for greenhouse tomatoes based on the real data set.	The experimental data were collected at the Xiaotangshan National Precision Agriculture Research and Demonstration Base’s tomato sunshine greenhouse in Beijing’s Changping District.	A water-saving irrigation decision-making algorithm based on genetic optimization T-S fuzzy neural network was developed to optimize greenhouse tomato irrigation water resource consumption.	We also used the revised genetic algorithm to tune the initial weights and thresholds of the T-S fuzzy neural network. Furthermore, using the real data set, we assessed the accuracy of the GA-TSFNN by simulating and predicting greenhouse tomato irrigation volume.	The optimization algorithm and constraint operators are not properly included, which is why it is required to be improved.
IoT-based model using Raspberry Pi (Krishna et al., 2017)	A unique wireless mobile robot based on the Internet of Things (IoT) is created and implemented to perform diverse field operations.	The various data are collected through all the sensors such as thermo hygro sensor, soil moisture, humidity, ultraviolet, CO_2_, ultrasonic, and pH.	This suggested wireless robot is outfitted with a variety of sensors that measure various environmental conditions. It also includes the Raspberry Pi 2 model B hardware for running the entire process. The major characteristics of this revolutionary intelligent wireless robot are that it can perform activities such as moisture detection, scaring birds and animals, spraying pesticides, moving forward or backward, and switching an electric motor ON/OFF.	It is outfitted with a variety of sensors to monitor various environmental conditions relevant to crop yield. Wireless crop monitoring reduces labor costs while also allowing for accurate tracking of changes that occur in real time in the field.	The construction of this model is not always friendly to the environment and is expensive.
IoT and Big Data-enabled self-driven model (Keswani et al., 2020)	This research focuses on the efficient control of farm irrigation by leveraging the capabilities of the Internet of Things (IoT) and Big Data-based decision support system (DSS) to generate appropriate valve control orders.	The proposed IoT node deployment approach, which has been field-tested, is used to capture real-time data.	An integrated IoT-based DSS framework is suggested to collect 17 soil and ambient characteristics in order to forecast future changes in soil moisture levels in 1 h.	Irrigation regulation by zone and crop is a key responsibility in all agricultural fields. The suggested IoT deployment framework has been thoroughly tested in the field to obtain uniform soil moisture levels throughout the target crop-specific zones.	The irrigation system is not all climate-supported, which means it needs to be improved.

In **Table 7**, we can see how the 5G network stacks up against other existing network generations. High-definition video streaming and telephony were made possible on the road by 4G networks, an improvement above 3G. As network traffic has increased, the theoretical maximum for 4G speeds has been reached. According to the ITU, the most recent 5G use cases fall into one of three categories: ultrareliable low latency communications (URLLC), massive machine type communications (mMTC), and enhanced mobile broadband (eMBB).

**Table 7:** Comparison of the proposed generation of network with existing networks.

Parameters	2G	3G	4G	5G (proposed network)
Year of launching	1993	2001	2009	2018
Technology	GSM	WCDMA	LTE, WiMAX	MIMO, mmWaves
Active system	TDMA, CDMA	CDMA	CDMA	OFDM, BDMA
Switching type	Circuit, packet	Circuit, packet	Packet	Packet
Network	PSTN	PSTN	Packet network	Internet
Internet access	Narrowband	Broadband	Ultra broadband	Connectionless World Wide Web
Bandwidth	25 MHz	25 MHz	150 MHz	30–300 GHz
Speed	64 Kbps	8 Mbps	300 Mbps	10–30 Gbps
Latency	300–100 ms	100–500 ms	20–30 ms	1–10 ms
Mobility	60 km	100 km	200 km	500 km

**Table 8** shows that Odisha is in the fifth position all over India. This table shows only the seasonal production of tomatoes in India. If the display of tomatoes is required to produce in non-seasonal duration (August to October), then the state Odisha is considered in the third position. The implementation of the intelligent cultivation method improves the situation in the production table.

**Table 8:** Tomato production details in India.

	States	Production qty (M tons)	Share (%)	
1	Andhra Pradesh	2,744	13.9	Major tomato production state in India
2	Madhy Pradesh	2,419	12.2	
3	Karnataka	2,081	10.5	
4	Gujurat	1,357	6.9	
5	Odisha	1,312	6.5	
6	West Bengal	1,265	6.4	
7	Telegana	1,171	5.9	
8	Telegana	1,087	5.5	

**Table 9** shows the exportation of tomatoes from India to other countries. The export is done in the seasonal duration of production, but it is required to export in a non-seasonal period through intelligent irrigation techniques. **Table 10** shows the importation of tomatoes to India in the case of seasonal duration. The IoT-based intelligent irrigation method provides a technique to cultivate tomatoes in the non-seasonal period, so that there is no need to import from outside of the country, which gives better performance than the traditional cultivation process.

**Table 9:** Exportation of tomatoes from India to other countries.

	States	Production qty (M tons)	Values (million US $)
1	U ARAB EMTS	32,172.6	16.33
2	Qatar	14,309.6	8.32
3	Singapore	102.74	0.12
4	Malaysia	100.99	0.06
5	Saudi	96.22	0.05
6	Austria	14.65	0.03

**Table 10:** Importation of tomatoes from other countries to India.

	States	Production qty (M tons)	Values (million US $)
1	China	15,213	12.74
2	USA	3,028	3.01
3	Spain	1,248	1.06
4	Italy	796	0.11
5	Chile	115	0.05
6	Bhutan	65	0.03

## 6 Conclusion with future work

In this approach, traditional fields such as agriculture require technology (here, smart farming) to achieve higher crop yields with less human intervention in a limited time frame. Smart farming, on the other hand, necessitates significant investment, improved coverage and connectivity, and more bandwidth to manage the massive amount of data generated by a huge number of sensors and equipment deployed remotely. Although the 4G network has a huge capacity and adequate coverage, it is unable to transmit the massive amount of real-time data between a large number of devices. The introduction of 5G meets current criteria and demands in smart farming to boost output with minimal human effort. Thus, the production of tomatoes mostly suffers due to improper management of moisture levels and irrigation.

To overcome this problem, a smart irrigation system was proposed by using the IoT framework. The required moisture levels and the amount of water were predicted to improve the production of tomato yield. IoT modules were used to optimally evaluate the requirement for water amount and smartly process the irrigation system. A mobile application was also developed that can help farmers by providing useful information. Extensive experimental results indicated that the proposed model can smartly optimize the irrigation system which helps to improve tomato production. Based on the simulation results and analyses of previously stored data, our platform could be used to generate important analytics of real-time monitoring, enabling decisions and actions like managing the irrigation system or building alters, for example. Throughout our trial, we have only encountered a few restrictions, such as the need for a reliable power source and wireless connectivity to communicate with the cloud. A comparison of the proposed model and other existing networks was included in the manuscript as shown in **Table 6**.

In the near future, we will implement the proposed framework for other crops. Additionally, we will evaluate the suggested framework in a simulated environment by combining the nodes and transferring data based on criteria such as lifetime, throughput, and latency. More application-specific case studies would be helpful in tailoring the general framework for QoS assurance.

## Data availability statement

The original contributions presented in the study are included in the article/Supplementary Material. Further inquiries can be directed to the corresponding author.

## Author contributions

DSi and AB: conceptualization. DSa and VS: methodology. SK and AK: software and validation. YN: supervision. All authors contributed to the article and approved the submitted version.
